# Prediction of Research Hotspots Based on LSTM: Taking Information Science as Example

**DOI:** 10.1155/2022/2849815

**Published:** 2022-06-25

**Authors:** Fuzhong Xiang

**Affiliations:** Institute of Information Management, Shandong University of Technology, Zibo, Shandong 255000, China

## Abstract

Detection and identification become the prediction of future research hotspots in the discipline, which is important to grasp the current status and development trend of the discipline research. In this paper, we use the cumulative topic heat model to calculate the research heat of each research topic in intelligence science from 2000 to 2020 and use the first 70% of the data as the training set, use the LSTM model for prediction, and construct the ECM model for error correction. The actual topic hotness of intelligence science for the latter 30% of data was used as the validation set to verify the effectiveness of the method. It was found that the average deviation rate of the method's prediction results fluctuated between 9.75% and 12.68%, and the average number of error entries was about 0.161, which had high validity. The study also predicts that by 2025, topics such as “crisis warning” and “health information services” in intelligence will continue to rise in popularity and “scientific data” and “data mining” will continue to rise in popularity. The hotness of “data mining” will remain stable, while the hotness of “citation analysis” and “ontology” will gradually decline.

## 1. Introduction

With the rapid development of science and technology and the national promotion of “new liberal arts construction,” the scientific research of intelligence science presents the characteristics of interdisciplinarity and high dynamics [1]. To grasp the historical research hotspots and the current research status of the discipline and to predict and analyze the future research direction of the discipline, it is helpful to assist management departments, research departments, and scholars to invest limited research resources in relevant research fields with high potential, which is of practical significance to promote the development of the discipline.

The long-term and short-term memory network—usually referred to only as “LSTM”—is a special RNN that can learn long-term rules. They were first proposed by Hochreiter and Schmidhuber (1997) and were refined and popularized by many people in later work. They are applied very well on various problems and are now widely used.

Academic journals are important carriers of knowledge, and keywords are the condensation of research topics of academic journal papers. Therefore, in this paper, the keywords of academic journals are used to represent the research topics of the papers, and the TP model of cumulative hotness of topics is used to calculate the research hotness of each topic in intelligence from 2000 to 2020. Among them, the first 70% of the data being the training set, i.e., the research hotness from 2000 to 2015, are substituted into the LSTM model for prediction, and the latter 30% of the data, i.e., the data from 2016 to 2020, are used as the validation set for the validity of the prediction results to verify the validity of the model.

## 2. Related Work

Disciplinary hotspots are highly popular research topics that are widely followed and studied by researchers, which are the key areas of disciplinary research and represent the future development direction of the discipline [2]. Disciplinary research hotspots are often dynamic and inherited and generally do not arise or disappear out of nowhere in a short period of time, which is a prerequisite for being able to conduct keyword-based analysis and prediction of disciplinary research hotspots [3]. Carrying out prediction research of disciplinary hotspots and grasping the dynamic changes and dominant trends of disciplinary research are of great guiding significance for the research and development, innovation, etc. of the discipline.

The prediction of future trends of research hotspots is carried out based on research hotspot identification methods, and scholars at home and abroad use different methods to identify disciplinary research hotspots. Currently, there are two major categories of methods in the identification of research hotspots and frontier hotspots in intelligence and science: citation analysis methods (e.g., co-citation and literature coupling) and text content analysis (word frequency analysis, co-word, and topic probability model analysis). Mane and Börner [4] used Kleinberg burst detection and co-word analysis to identify hotspots in the *Proceedings of the National Academy of Sciences of the United States of America*; Chang et al. [5] used citation coupling and co-citation analysis to identify research hotspots in library intelligence; Hu and Gao [6] used multiword co-occurrence and cluster analysis to identify hotspots in library intelligence strategic planning journals and successfully identified hotspots in domestic library strategic planning research; Qiu and Shao [7] proposed an LDA2vec model based on LDA and Word2Vec and successfully identified hotspots in multisource data environment for hotspot identification and demonstrated the feasibility of the method; Guohe Feng and Feng [8] revealed disciplinary research hotspots and changing trends by constructing a time-weighted keyword word frequency analysis model and verified the scientificity and effectiveness of the method by taking the research field of library intelligence as an example; Li et al. [9] identified intelligence research hotspots by improving the *Z* index and “successfully identified” Li et al. [9] successfully identified three different types of research trends, namely, “rising,” “stable,” and “declining,” by improving the Z-index; Chen et al. [10] used Bicomb, Ucinet, Citespace, and other software to predict the research trends in the field of clinical medicine in China; and Chen et al. [10] used Bicomb, Ucinet, Citespace, and other software to forecast and analyze the research hotspots and development trends in the field of clinical medicine research in China.

Scholars mostly construct prediction models by predicting disciplinary research hotspots. Liu et al. [3] successfully identified research hotspots by the prediction method of time series model, taking the field of competitive intelligence as the research object, and proved the effectiveness of the method; Ming and Xu [11] analyzed the core journals in the field of graphical intelligence in China by the association rule mining method of Apriori algorithm and made short-term predictions for four groups of typical keyword sets to analyze their future development trends; Guo and Wang [12] used co-occurrence analysis method and hierarchical clustering method to make hotspot prediction of domestic reading promotion research hotspots and predicted the development trend of class groups in the next three years with gray GM (1,1) model; Li et al. [13] used information visualization software Citespace to analyze literature in the field of patent infringement risk warning, predicted research hotspots and frontier trends, and put forward related topics such as intelligent warning analysis; Wen et al. [14] applied the statistical evolution trajectory prediction method to predict Chinese intelligence journal papers and identified some possible hot keywords in intelligence; and Yi et al. [15] used the LSTM hot spot prediction model to predict the hot spots of public opinion in colleges and universities and verified the accuracy of LSTM for predicting public opinion trends by comparing the two models of support vector machine and recurrent neural network.

In addition, some scholars have conducted research on the comparison of research hotspot prediction methods and models. It is found that the citation analysis methods based on co-citation and literature coupling have the lag of time detection, and the problems of not going deeper into the text content and lacking semantic relationships limit the scientificity of hot topic detection to a certain extent; the traditional time series prediction methods focus on mathematical statistics and do not have self-learning, self-organization, and self-adaptive capabilities, especially for nonlinear and multi-feature dimensional data. With the construction of Internet of everything and big data ecosystem, time series prediction models based on machine learning and deep learning algorithms are increasingly playing an important role. Li and Xu [16] used the genetic engineering field as the analyzed data source and used representative machine learning algorithms such as BP neural network, support vector machine, and LSTM model for hotspot trend prediction, and the research results showed that among the prediction methods of machine learning algorithms, LSTM model has the highest prediction accuracy and better stability, followed by support vector machine, and BP neural network is less stable.

In summary, researchers have actively explored the hotspot identification and prediction using many research methods. Compared with traditional citation analysis and text analysis identification and prediction methods, machine learning algorithms prediction models are increasingly playing an important role. However, in hotspot identification research using machine learning for prediction, scholars have mostly compared multiple prediction models, neglecting to correct for prediction errors, resulting in relatively low accuracy rates. In this paper, based on the LSTM model, the prediction results are corrected by constructing an error correction model to make the identification results more accurate and the prediction results more precise.

## 3. LSTM Model-Based Prediction Method

### 3.1. Research Method Design

The general research idea of this paper is shown in Figure 1.

In Figure 1, in this paper, after collecting sample question records and preprocessing, the data are divided into training set and test set, where the training set includes a total of 16 years of data from 2000 to 2015 and the test set includes a total of 5 years of data from 2016 to 2020. The main research ideas are as follows:

1. Measuring the cumulative topic hotness TP of the machine learning samples and grouping them to evaluate the research hotness of each topic in the historical data
2. Substituting the results of the cumulative topic hotness TP calculation of the above samples into the LSTM model for machine learning to predict the predicted TP values for 2016–2020
3. Calculating the actual TP values of the validation set and performing accuracy analysis between them and the predicted TP values, using the metrics of average deviation rate and average error value
4. If the validation result is that the prediction model is valid, the LSTM model is used for future trend prediction
5. The data patterns of the identification results are analyzed and classified according to the different characteristics of the future hot topics

### 3.2. Cumulative Heat Study

In this paper, we adopt the TP ∗ TAI model constructed by Rong et al. [17], which is able to measure the cumulative subject hotness TP model of the subject. The model uses a cumulative calculation to reflect the relative cumulative research hotness of a topic, i.e., the proportion of the cumulative word frequency (i.e., volume of research literature) of a research topic in the total disciplinary literature in a certain time period, which is given by

(1) $$\begin{array}{c} \text{TP}=\frac{\sum_{t=n}^{i}C_{t}}{\sum_{t=n}^{i}P_{t}},\;n\leq i\leq m. \end{array}$$

In equation (1), TP is the cumulative hotness of keywords, *t* is the year, *C*_*t*_ is the volume of research literature on a research topic in year *t*, and *P*_*t*_ is the total subject literature in year *t*. *n* is the year in which the subject term first appears or the starting year of data grouping, and *m* is the most recent year or the cut-off year of data grouping. TP model not only reflects the hotness of subject development up to year *t* but also eliminates the literature in each year. The TP model not only reflects the hotness of the topic development up to year *t* but also eliminates the theoretical error caused by the different absolute number of literature in each year.

### 3.3. Introduction of the LSTM Model

The long short-term memory network (LSTM) is a special RNN recurrent neural network model. The LSTM model has a long-term memory function, which is suitable for the prediction of time series and can solve the problem of gradient disappearance well [18]. Its basic principle is shown in Figure 2.

LSTM is based on RNN, the original tanh layer is improved to memory gate, and 2 neural network layers of forgetting gate and cell state are added to the original output gate. The roles and basic principles of the 4 neural network layers of the model are as follows:

(1) The forgetting gate plays the role of data screening, i.e., deciding which information to keep and which information not to keep. The expression of its basic principle is as follows:
  (2) $$\begin{array}{c} f_{t}=\sigma \left(W_{f}\cdot \left[h_{t-1},x_{t}\right]+b_{f}\right). \end{array}$$
In equation (2), *h*_*t*−1_ and *x*_*t*_ denote the data inherited from the previous state. They are operated with the forgetting gate weight *w*_*f*_ and the bias constant *b*_*f*_ is introduced. When the value of *f*_*t*_ is infinitely close to 1, the program chooses to keep the data; when the value of *f*_*t*_ is infinitely close to 0, the program chooses to delete the data.
(2) The memory gate plays the role of data storage, i.e., inputting information into the new cell state. The expression of its basic principle is as follows:
  (3) $$\begin{array}{c} i_{t}=\sigma \left(W_{i}\cdot \left[h_{t-1},x_{t}\right]+b_{i}\right),\\ D_{t}=\tanh\left(W_{d}\cdot \left[h_{t-1},x_{t}\right]+b_{d}\right). \end{array}$$
(3) Updating the cell state is the process of data integration. The new cell state *C*_*t*_ is obtained by adding the data obtained from the forgetting gate and the data obtained from the memory gate based on the obtained data. The new *C*_*t*_ contains the data to be discarded and the new data to be added, which is passed into the next LSTM model.
  (4) $$\begin{array}{c} C_{t}=f_{t}\times C_{t-1}+i_{t}\times D_{t}. \end{array}$$
Equation (5) combines the data from the forgetting gate and the memory gate to update the cell state *C*_*t*_.
(4) The output gate plays the role of transferring the machine learning data and outputting the prediction results.
  (5) $$\begin{array}{c} E_{t}=\sigma \left(W_{E}\left[h_{t-1},x_{t}\right]+b_{E}\right), \end{array}$$
  (6) $$\begin{array}{c} h_{t}=E_{t}\times \;\tanh\left(C_{t}\right). \end{array}$$

In Equation (6), *E*_*t*_ is responsible for controlling the output long-term memory. Equation (7) is responsible for the output of the final prediction *h*_*t*_.

(7) $$\begin{array}{c} \text{ECM}=\Delta Y=\frac{C_{1}}{P_{1}}\Delta X+0.0014\text{ecm}\left(t-1\right)-\frac{C_{t}}{P_{t}}t. \end{array}$$

### 3.4. Error-Corrected ECM Model Construction

Although the topic cumulative hotness model TP has the theoretical feasibility of substitution into the LSTM model, direct substitution may generate large errors because the TP Model is not designed for neural network models. Therefore, equation (1) is processed by the difference method to reduce the influence of time on the data, thus eliminating the dependence of the data on time. The transformation results are

(8) $$\begin{array}{c} Y_{t}=\alpha_{i}X_{t};\alpha_{i}=\frac{\sum^{}C_{i}}{\sum^{}P_{i}},\;i\in \left[n,m\right],\alpha_{i}\in \left(0,1\right], \end{array}$$

where *c*_*i*_ and *p*_*i*_ are the predicted and actual values in the time slice, respectively, and *X*_*t*_ is the actual average value during the observation time. For the whole discipline, *X* and *Y* are rarely located at the equilibrium point alone, so what is actually observed is only a short-term disequilibrium relationship, assuming a lagged form with a (1, 1) order distribution, it can be found that the change in *Y* in period *t* depends not only on the change in *X* itself but also on the state of *X* and *Y* at the end of period *t* − 1, so the simple difference does not necessarily solve all the problems encountered in a smooth time series, so it is necessary to further introduce the error correction model.

In order to obtain more accurate hotness prediction results and to classify hotspots more precisely using the slope *K* of the regression equation, this paper introduces an error correction model (ECM) to correct the results based on zero-sum game theory (Zero-sum Game) and the broken window effect (Break Pane Law). Considering that in future practical research, the TP values we obtained for the subject keywords may be under nonstationary time series, we try to avoid using the OLS method to establish the ECM and the transformation of equation (9) is obtained as follows:

(9) $$\begin{array}{c} \Delta Y_{t}=\beta_{i}\Delta X_{t}-\lambda \left(Y_{t-1}-\alpha_{i}X_{t-1}\right)+\varepsilon_{t},\\ \lambda =1-\mu ,\\ \alpha_{i}=\frac{\beta_{i}+\beta_{i+1}}{1-\mu }, \end{array}$$

where *μ* and *β*_*i*_ are the slope of the predicted value per unit of time and the linear intercept between the actual and predicted values, respectively. Equation (10) shows that the change in *Y* is determined by the change in *X* and the degree of disequilibrium in the previous period, to make up for the shortcomings of the simple difference model through the degree of disequilibrium in the previous period, when the *Y* value of the degree of disequilibrium in the previous period has been made to correct, so (9) formula is also known as the first-order down error correction model, according to which the (9) formula can be changed to

(10) $$\begin{array}{c} \Delta Y_{t}=\beta_{1}\Delta X_{t}-\lambda \text{ecm}+\varepsilon_{t}, \end{array}$$

where ecm denotes the error correction term, and the distribution lag model knows that in general there is |*μ*| < 1; 0 < *λ* < 1; at this time, the correction effect of ecm is as follows: when (*t* − 1) when *Y* > equilibrium solution, ecm > 0, and (−*λ*ecm) < 0, so that Δ*Y*_*t*_ ↓, at this time *β*_*i*_ can be regarded as the short-term elasticity of *Y* with respect to *X*; after calculation, the final error correction model ECM is obtained as

(11) $$\begin{array}{c} \text{ECM}=\Delta Y=\frac{C_{1}}{P_{1}}\Delta X+0.0014\text{ecm}\left(t-1\right)-\frac{C_{t}}{P_{t}}t. \end{array}$$

## 4. Empirical Study: Intelligence as an Example

### 4.1. Data Source and Preprocessing

In this paper, taking intelligence as an example, the sample is selected based on the top ten CSSCI source journals in terms of CNKI's comprehensive impact factor ranking in 2020. Since the data of Journal of Intelligence from 2003 to 2012 were not included in the database of Zhiwang, the collected data were missing part of the literature of *Journal of Intelligence* and could not be used as the research sample. Therefore, the research samples finally selected in this paper are *Chinese Library Journal*, *Library and Intelligence Work*, *Library and Intelligence Knowledge*, *University Library Journal*, *Book and Intelligence, Intelligence Theory and Practice, Intelligence Information Work*, *Intelligence Science, and Journal of Intelligence*, a total of nine. Using the Zhiwang database as the data source, a scripting program was written to collect the title data of a total of 53,228 documents from 2000 to 2020 from the above journals and deposit them into the MySQL database.

The above data were preprocessed according to the following steps:

1. Remove 2011 nonresearch papers such as volume headings, editorial announcements, and submission notes to obtain a valid sample data of 51217 papers and deposit the sample data into the MySQL database.
2. Write a PHP program to split, count, and output the keywords in the title list information.
3. Data cleaning and synonym merging. We screened out the words that indicated the background of the study, such as “America” and “China,” as well as the words with unknown meanings that could not indicate the content of the study, such as “influence factors” and “empirical study.” “Merge keywords with the same meaning, such as “HMM” and “Hidden Markov Model,” into “Hidden Markov Model,” etc.

### 4.2. Cumulative Hotness TP Model Calculation

In this paper, the data are processed according to the following steps:

1. Write a PHP program to extract high-frequency keyword word frequency *C*_*t*_ from MySQL database, count its word frequency, and count the total number of articles issued each year *P*_*t*_. Set the threshold value of keyword word frequency as 5, extract 1359 high-frequency keywords in intelligence science, and count *C*_*t*_, *P*_*t*_, respectively, year by year. The statistical results are shown in Table 1. In Table 1, information management: is the management of information resources and information activities; search engine: “the so-called search engine” is based on user needs and certain algorithms, using a specific strategy to retrieve specified information from the Internet back to the user of a search technology; in the World Wide Web: to disseminate, exchange, service in the field of resource science comprehensive, or subspecialty information hypertext transfer HTTP (Hypertext Transfer Protocol) server, which provides a set of associated HTML (Hypertext Markup Language) resource information documents, and related documents, processes, and databases; Intellectual property rights: “a collective term for the rights that arise under the law based on creative works and industrial and commercial marks.” The three main types of intellectual property rights are copyrights, patents, and trademarks, of which patents and trademarks are also collectively referred to as industrial property rights.
2. Cumulative topic hotness TP calculation. *C*_*t*_ and *P*_*t*_ were substituted into formula (1) year by year to obtain the TP values of topic hotness, as shown in Table 2. Among them, in order to avoid the cumulative hotness calculation where the new increment is much smaller than the cumulative amount leading to the accumulation of too large denominator of the model and losing the effect of measuring the topic hotness, the data are grouped, i.e., every 5 years as a group (the TP value of 2020 is calculated separately), and the TP value is calculated. The calculation results are shown in Table 2.

### 4.3. LSTM and ECM Model Validity Analysis

#### 4.3.1. Cross-Sectional Comparison of Prediction Models

In order to verify the prediction effectiveness of LSTM model, this paper adopts a cross-sectional comparison approach and selects four prediction models, SVM, RNN, linear regression, and BP neural network, which are used more frequently and widely recognized, for comparison with the LSTM prediction model. The deviation rate calculation formula is introduced, and a sampling approach is taken to measure the deviation rate of the data with the measured results and after the ECM intervention. The time range of the measurement is chosen for the validation set, i.e., 2016–2020, and then the average of the 5-year deviation is measured as the average prediction deviation rate. The deviation rate MD for individual years is calculated as follows:

(12) $$\begin{array}{c} \text{MD}=\frac{\left|P_{r}-T_{r}\right|}{T_{r}}, \end{array}$$

where *P*_*r*_ is the predicted TP value and *T*_*r*_ is the actual TP value. From the results of each prediction model, 300 results were randomly selected from each model, and the average deviation rate before and after ECM intervention was calculated. The results are shown in Table 3.

According to Table 3, the deviation rate of LSTM is relatively low compared with the other four prediction methods. Therefore, it is reasonable to choose the LSTM model as the main prediction method in this paper.

#### 4.3.2. ECM Model Validity Analysis

The calculated TP values from 2000 to 2015 in Table 1 are used as the training set for the LSTM model, and the error correction is performed using equation (11). Python 3.9 is used as the running environment, and a self-programmed program is used to process the data. The program first reads the existing data and then calculates the existing data line by line using LSTM model. The predicted values of the 2016–2020 data are obtained. In this paper, we take the 2020 data as an example to show the effect of LSTM prediction and the effect of ECM model intervention, as shown in Table 4.

In Table 4, the 2016–2020 data are used as the validation set of this prediction model, in which the average correction after the intervention of the ECM error correction model is around 51.56%, indicating that the error correction model derived in this paper can better reduce the error of the LSTM prediction of the cumulative topic hotness TP Model. Therefore, this paper uses the data after ECM intervention as the final prediction result for LSTM model validity analysis.

#### 4.3.3. Average Deviation Rate Measure of Prediction Results

In order to ensure the accuracy of the prediction results, the prediction results of the validation set were sampled several times to avoid the chance of word sampling results. Totally, 300 keyword data are randomly selected from the validation set for deviation rate calculation, and the above process is repeated five times. The results of the five sampling times are shown in Table 5.

In Table 5, the maximum average deviation rate is 13.68% and the minimum average deviation rate is 8.42% after five random sampling. This indicates that the average deviation rate of the prediction results is low and the prediction results have validity.

#### 4.3.4. Estimation of the Actual Average Number of Errors

The average error value is measured between the predicted and actual values of LSTM in 2020. The measurement method is as follows: the predicted value of cumulative hotness TP of all data is subtracted from the sum of the absolute values of the actual values and divided by the total number of keywords to obtain the average error value of all data *A*. The formula is as follows:

(13) $$\begin{array}{c} A=\frac{\sum_{i=1}^{K}\left|{\text{TP}}_{i}-{\text{TP}}_{pi}\right|}{K}, \end{array}$$

where TP_*i*_ represents the actual TP value of the *i*th keyword, TP_*pi*_ represents the predicted TP value after ECM intervention for the *i*th keyword, and *K* represents the total number of keywords. Substituting columns 2 and 3 in Table 4 into the average error value calculation formula (14), we get

(14) $$\begin{array}{c} A=\frac{\sum_{i=1}^{K}\left|{\text{TP}}_{i}-{\text{TP}}_{pi}\right|}{K}=\frac{0.544}{1359}=0.0004. \end{array}$$

In order to make the results look more intuitive, this paper converts the average error TP value into the actual number of error articles, i.e., the average actual word frequency value of each keyword minus the predicted word frequency value. The conversion process and the results are as follows:

(15) $$\begin{array}{c} C_{2020}-C_{p2020}=\left|\left({\text{TP}}_{2020}\times P_{2020}\right)-\left({\text{TP}}_{P2020}\times P_{P2020}\right)\right|\\ =\left|0.000129\times 10075-0.000145\times 10075\right|=0.161. \end{array}$$

According to the above calculation results, it can be seen that in 2020, the average error between the predicted and actual number of articles per research hotspot is 0.161, which indicates that the prediction results have some validity.

### 4.4. Analysis of Prediction Results

#### 4.4.1. Calculation of Predicted TP Values

Based on the validation of the validity of the method in this paper, the TP calculation results in Table 1 are substituted into the LSTM model for prediction, the ECM model is used for correction to predict the TP of the topic hotness of keywords in 2021–2025, and the prediction results are displayed in Table 6.

#### 4.4.2. Basis for the Classification of Topic Prediction Results

The prediction results in Table 4 can reflect the future research hotness of topic terms and their changes. In this paper, the topic prediction results are classified into rising, stable, and falling according to the slope of change of the cumulative topic hotness TP.

The regression equation of TP prediction value is generated using a self-programmed program in Python, and the proposed division is based on the following: (1) ascending research hotspot, i.e., the future probability of maintaining an upward trend of hotness, with a slope greater than 1; (2) stable research hotspot, i.e., the future probability of continuing to fluctuate to maintain an upward or stable state, with a slope between −1 and 1, the closer to 0, the more stable the fluctuation; (3) declining research hotspot, i.e., the future probability of continuing to fluctuate to maintain an upward or stable state. That is, the future probability of hot continues to decrease, the slope is less than −1. The slope of the regression equation of some keywords is shown in Table 7.

In addition, the LSTM model is found to be less effective in predicting research hotspots that are more emergent, such as “novel coronary pneumonia” and “public health emergencies.”

A VBA program is written to classify the themes into future rising, stable, and declining according to the theme classification basis, which is displayed in Table 8.

#### 4.4.3. Analysis of Future Research Hotspots

According to the prediction results of this paper, the development trend of future intelligence research hotspots is analyzed:

1. Rising research hotspots are characterized by a high proportion of research hotness and a fast growth rate and have greater potential and development momentum in the next few years. Among them, in the context of the normalized prevention and control of the new pneumonia epidemic, intelligence research on crisis warning and health information services ranks among the top two “rising” research hotspots and mostly focuses on the study of network rumor crisis warning [19], epidemic network public opinion warning [20], and microblog public opinion warning [21].
2. Stable research hotspots are characterized by relatively stable hotness on the macro level and fluctuating development on the micro level, which are the core research contents of intelligence science and will probably maintain their research hotness in the next few years. Among them, social network analysis is the process of investigating social structure through the use of networks and graph theory, which characterizes the network structure in terms of nodes (individuals, people, or things in the network) and the ties, edges or links that connect them, providing a method for qualitatively assessing networks [22]. In recent years, social network analysis methods have been combined with theoretical approaches in intelligence, mostly for intelligence analysis [23–25], opinion dissemination [26], and co-authorship network research [27]. The research contents of bibliometrics and data mining, on the other hand, belong to the more stable core research directions of intelligence, and in recent years, they mainly focus on research hotspot identification [28], interdisciplinary knowledge flow [29], topic evolution [30], knowledge mapping [31], etc.
3. Declining research hotspots will probably decline in hotness in the next few years, indicating that such topics have accumulated certain research results in the development process and have developed relatively mature, and will undergo topic evolution, more in-depth and detailed research, or shift to similar research fields in the future [32].

## 5. Conclusion

In this paper, we first calculated the research hotspot degree of each research topic in the field of intelligence from 2000 to 2020 by using the TP model of cumulative topic hotspot, divided the data into training and validation sets, and constructed an error correction ECM model. Next, the LSTM model was compared with other prediction models in cross section to verify the rationality of using the LSTM model. Then, the average deviation rate and average deviation value are calculated from the LSTM prediction TP values to the validation set to verify the validity of the model in this paper. Finally, the predictions of intelligence research hotspots for 2021–2025 were divided into three categories: “rising,” “stable,” and “falling.” However, recent hot topics such as “new crown pneumonia” only use the horizontal cumulative word frequency ratio to reflect the hotness of the topic, which is a single measure. This will be the direction of our future efforts.

## Figures and Tables

**Figure 1:** Overall research idea diagram.

**Figure 2:** Schematic diagram of the LSTM model.

**Table 1:** *C*_*t*_ and *P*_*t*_ statistics results (partial).

Keywords	2000	2001	2002	2003	2004	2005	2006	2007	2008	2009	2010	2011	2012	2013	2014	2015	2016	2017	2018	2019	2020
Information management	25	32	29	24	22	27	18	31	9	18	13	10	9	11	8	4	8	10	2	5	4
Search engine	24	35	39	33	28	39	28	21	11	16	14	11	13	11	7	7	6	4	2	3	1
Intelligence	23	29	33	40	40	61	43	55	56	67	34	58	48	36	43	32	22	34	23	27	29
Librarian	23	23	27	17	29	12	21	15	13	12	17	13	14	12	9	10	15	5	4	4	3
Enterprise	22	24	27	13	34	33	27	29	22	29	54	41	37	21	21	15	13	12	13	8	3
Web information resources	18	23	25	32	35	22	18	12	13	15	7	5	16	3	7	4	2	3	1	1	1
Library automation	18	17	14	3	2	1	2	0	0	0	1	0	0	1	0	2	1	0	0	0	0
Documentary pnformation	18	8	13	4	10	4	3	1	3	0	1	3	0	1	0	0	0	0	0	1	1
Library management	18	29	41	34	41	29	20	15	14	8	18	9	7	5	3	4	1	0	3	1	0
Intellectual property	18	16	38	26	43	12	30	18	12	24	20	25	14	9	8	5	4	1	9	7	3
…	…	…	…	…	…	…	…	…	…	…	…	…	…	…	…	…	…	…	…	…	…
*P*_*t*_	1786	2414	4973	7342	10042	12626	2702	5224	7720	10843	14159	3352	6235	8791	11221	13512	2195	4250	6202	8096	10075

**Table 2:** Cumulative hotness TP calculation results (partial).

Keywords	2000	2001	2002	2003	2004	2005	2006	2007	2008	2009	2010	2011	2012	2013	2014	2015	2016	2017	2018	2019	2020
Information management	0.014	0.013	0.012	0.012	0.011	0.011	0.007	0.009	0.008	0.007	0.006	0.003	0.003	0.003	0.003	0.003	0.004	0.004	0.003	0.003	0.003
Search engine	0.013	0.014	0.015	0.015	0.013	0.014	0.010	0.009	0.008	0.007	0.006	0.003	0.004	0.004	0.004	0.004	0.003	0.002	0.002	0.002	0.002
Intelligence	0.013	0.012	0.012	0.014	0.014	0.016	0.016	0.019	0.020	0.020	0.018	0.017	0.017	0.016	0.016	0.016	0.010	0.013	0.013	0.013	0.013
Librarians	0.013	0.010	0.010	0.009	0.010	0.009	0.008	0.007	0.006	0.006	0.006	0.004	0.004	0.004	0.004	0.004	0.007	0.005	0.004	0.003	0.003
Enterprise	0.012	0.010	0.010	0.009	0.010	0.010	0.010	0.011	0.010	0.010	0.011	0.012	0.013	0.011	0.011	0.010	0.006	0.006	0.006	0.006	0.005
Web information resources	0.010	0.010	0.010	0.011	0.011	0.011	0.007	0.006	0.006	0.005	0.005	0.001	0.003	0.003	0.003	0.003	0.001	0.001	0.001	0.001	0.001
Library automation	0.010	0.007	0.006	0.005	0.004	0.003	0.001	0.000	0.000	0.000	0.000	0.000	0.000	0.000	0.000	0.000	0.000	0.000	0.000	0.000	0.000
Documentary information	0.010	0.003	0.004	0.003	0.003	0.003	0.001	0.001	0.001	0.001	0.001	0.001	0.000	0.000	0.000	0.000	0.000	0.000	0.000	0.000	0.000
Library management	0.010	0.012	0.014	0.014	0.014	0.014	0.007	0.007	0.006	0.005	0.005	0.003	0.003	0.002	0.002	0.002	0.000	0.000	0.001	0.001	0.000
Intellectual property	0.010	0.007	0.011	0.011	0.012	0.011	0.011	0.009	0.008	0.008	0.007	0.007	0.006	0.005	0.005	0.005	0.002	0.001	0.002	0.003	0.003
…	…	…	…	…	…	…	…	…	…	…	…	…	…	…	…	…	…	…	…	…	…

**Table 3:** Comparison of different prediction methods with LSTM.

Prediction method	Average forecast deviation rate (%)	Average prediction deviation rate after ECM intervention (%)
SVM	22.435	16.366
RNN	19.911	17.843
Linear regression	28.572	26.767
BP neural network	19.322	15.377
LSTM	16.184	11.714

**Table 4:** LSTM model projections for 2016–2020 data (partial).

Keywords	LSTM prediction results (before ECM intervention) LSTM prediction results (after ECM intervention)					LSTM prediction results (before ECM intervention) LSTM prediction results (after ECM intervention)					Error correction rate
	2016	2017	2018	2019	2020	2016	2017	2018	2019	2020	
Libraries	0.0363	0.0432	0.0316	0.0286	0.0363	0.0389	0.0409	0.0346	0.0301	0.0347	46.7%
Digital library	0.0088	0.0082	0.0123	0.0116	0.0084	0.0104	0.0089	0.0119	0.0106	0.0089	55.6%
Information services	0.0098	0.0112	0.0108	0.0105	0.0091	0.0101	0.0106	0.0105	0.0095	0.0085	44.9%
Network environment	0.0010	0.0008	0.0010	0.0009	0.0007	0.0010	0.0008	0.0009	0.0008	0.0006	51.7%
Information resources	0.0022	0.0035	0.0041	0.0026	0.0032	0.0021	0.0032	0.0036	0.0028	0.0027	56.7%
Databases	0.0008	0.0007	0.0007	0.0005	0.0008	0.0008	0.0008	0.0008	0.0006	0.0008	36.4%
Librarianship	0.0033	0.0058	0.0065	0.0075	0.0065	0.0035	0.0051	0.0056	0.0071	0.0060	65.3%
E-commerce	0.0026	0.0017	0.0016	0.0013	0.0013	0.0028	0.0018	0.0017	0.0014	0.0014	53.0%
Knowledge management	0.0101	0.0102	0.0068	0.0066	0.0074	0.0098	0.0095	0.0078	0.0068	0.0068	48.0%
Information retrieval	0.0051	0.0060	0.0038	0.0043	0.0037	0.0057	0.0053	0.0042	0.0041	0.0035	57.3%
…	…	…	…	…	…	…	…	…	…	…	…

**Table 5:** Average deviation rate between predicted and actual values of LSTM.

Number of sampling times	Number of samples taken	Average deviation rate (%)
1	300	13.68
2	300	10.71
3	300	11.24
4	300	8.42
5	300	9.75

**Table 6:** Keyword hotness prediction results for 2021–2025 after ECM intervention (partial).

Keywords	2021	2022	2023	2024	2025
Digital library	0.009	0.007	0.003	0.000	0.007
Information resources	0.003	0.004	0.003	0.003	0.002
network	0.001	0.001	0.002	0.001	0.002
network environment	0.000	0.000	0.000	0.000	0.000
Internet	0.000	0.000	0.000	0.000	0.000
Databases	0.001	0.001	0.001	0.001	0.001
Resource sharing	0.002	0.002	0.002	0.002	0.002
Librarianship	0.005	0.001	0.004	0.008	0.006
Competitive intelligence	0.009	0.010	0.008	0.009	0.012
Knowledge management	0.004	0.003	0.005	0.009	0.000
…	…	…	…	…	…

**Table 7:** Slope of regression equation for hotspots in library intelligence research.

Keywords	Slope
Crisis alert	19.818
Industrialization	14.964
Health information services	12.991
Mobile services	12.418
NSTL	9.018
Big data	7.555
Knowledge graph	5.709
Information quality	5.318
…	…
Scientific data	0.418
Social network analysis	0.373
Scientific data	0.236
Literature measurement	0.182
Co-term analysis	−0.118
Data mining	−0.155
Intelligence studies	−0.191
Internet public opinion	−0.300
…	…
Ontology	−1.455
Citation analysis	−1.636
United States	−1.842
Library	−2.573
Information services	−2.909
E-commerce	−3.010
Intellectual property	−3.152
Artificial intelligence	−3.376

**Table 8:** Sudden, rising, stable, and declining research hotspots in library intelligence.

Type research	Hotspot
Rising	Upside crisis warning, health information services, industrialization, mobile services, NSTL, big data, knowledge graphs, information quality

Stable	Scientific data, social network analysis, bibliometrics, co-word analysis, data mining, intelligence, online public opinion

Declining	Ontology, citation analysis, libraries, information services, E-commerce, intellectual property, artificial intelligence

## Data Availability

The experimental data used to support the findings of this study are available from the author upon request.
